# The Establishment of Risk Evaluation Index System for Small- and Medium-Sized Agency Bookkeeping Companies

**DOI:** 10.1155/2022/8701591

**Published:** 2022-08-13

**Authors:** Qingfu Wu, Xiaoqian Zhang

**Affiliations:** Guangzhou Huashang College, Guangzhou, China

## Abstract

In recent years, China's economy has developed rapidly; many small companies have risen rapidly; and the tax system has become more and more standardized. Because many small businesses cannot afford to hire full-time accountants, they opt to outsource accounting services, giving small- and medium-sized bookkeeping firms a large market space. However, these opportunities also bring huge operational risks to small- and medium-sized bookkeeping companies. The purpose of this research is to help such enterprises carry out risk management and reduce operational risks. This study uses an analytic hierarchy process and a fuzzy comprehensive assessment approach to successfully combine quantitative and qualitative analysis and create a multilevel analysis structure model of the risk management evaluation index system of small- and medium-sized agency accounting firms. The structural model is verified by a case, the specific risk score of each factor is calculated through the scores of 20 experts, and the importance of risk is judged according to the size of the score, indicating that the structural model is feasible.

## 1. Introduction

In order to promote the healthy development of the agency bookkeeping industry, the “Administrative Measures for Agency Bookkeeping” was officially implemented in May 2016, which once again standardized the institutional management of the agency bookkeeping industry [1], but this did not fundamentally solve the problem of industrial development. The Financial Accounting (2018) No. 32 document particularly emphasized the need to strictly manage agency bookkeeping institutions, establish and improve the integrity incentive and untrustworthy punishment mechanism for the agency bookkeeping industry, and regulate the management of industry associations [2]. In March 2019, the Ministry of Finance issued relevant regulations to simplify the application materials for agency bookkeeping qualifications, shorten the statutory approval time limit, and stimulate the vitality of market entities [3]. The bookkeeping industry has experienced nearly 30 years of development, from the traditional manual mode to the computerized mode [4]. Due to the development of artificial intelligence, the accounting and taxation of agency bookkeeping companies have gradually become intelligent [5], which has brought greater influence to small- and medium-sized bookkeeping companies, and the problem of risk management has become increasingly prominent [6].

## 2. Methodology

### 2.1. Basic Method Theory

In the “Comprehensive Risk Management Framework” released by COSO in 2003, comprehensive risk management includes three dimensions [7] as shown in Figure 1.

The basic process of comprehensive risk management is divided into five steps. The implementation of risk management is inseparable from the communication of information [8]. Therefore, a complete risk management information system must be established [9], as shown in Figure 2.

The formation process of agency bookkeeping risk: risk event—risk taker—risk loss [10], as shown in Figure 3.

### 2.2. Choice of Risk Assessment Method

Risk assessment mainly refers to the qualitative or quantitative analysis of the probability and impact of risk events [11]. This research mainly adopts the analytic hierarchy process and the fuzzy comprehensive evaluation method to quantitatively analyze the risk of the agency bookkeeping company [12].

#### 2.2.1. AHP

AHP is an analysis method based on hierarchical decision-making [13]. For unstructured and relatively complex decisions [14], the use of AHP will greatly reduce the amount of engineering [15].

The specific steps of AHP are as follows: (1) constructing the index system, (2) constructing the judgment matrix, (3) calculating the hierarchical weight [16], (4) checking the consistency of each layer, (5) calculating the combined weight, (6) total consistency test, and (7) determining the weight as shown in Figure 4.

#### 2.2.2. Fuzzy Comprehensive Evaluation Method

The fuzzy comprehensive evaluation method is a comprehensive evaluation method that transforms qualitative evaluation into quantitative evaluation through the membership degree theory of fuzzy mathematics [17].

The specific steps of the fuzzy comprehensive evaluation method are [18]: (1) determining the evaluation object, (2) establishing the index system, (3) determining the evaluation set, (4) determining the index weight, (5) fuzzy comprehensive evaluation, and (6) analysis of the evaluation results as shown in Figure 5.

## 3. Establishment of the Risk Evaluation Index System for Small- and Medium-Sized Agency Bookkeeping Companies

### 3.1. Establishment of the Risk Assessment Index System

In practical applications, there are many types of risk factor identification methods [19], mainly including the following: (1) brainstorming method, (2) analysis process method [20], (3) analysis of relevant scenarios, (4) risk decomposition method [21], and (5) editing event tree method [22]. According to the actual situation of small- and medium-sized agency bookkeeping companies, this paper adopts the brainstorming method to identify the risk factors of these companies.

Organized and sent 20 experts to conduct in-depth research on small- and medium-sized bookkeeping companies. Through the discussion, summarize the main risks in five aspects: policy and legal risk, industry competition risk, information technology risk, undertaking business risk, and practitioner risk [23]. In the case of ensuring the comprehensiveness of the risk evaluation system, the risk evaluation index system in Table 1 is summarized and determined [24].

### 3.2. Establishment of Risk Assessment Set

In order to make the evaluation effect clearer, the evaluation using gradients within a range of the evaluated risk factors is usually adopted [25]. Five different continuous grade categories are selected for the agency bookkeeping risk evaluation set, and the five evaluation results are “no risk,” “small risk,” “average risk,” “high risk,” and “huge risk,” Specifically, it is represented by V = {V1, V2, V3, V4, V5}, in which the five evaluation results are, respectively, corresponding to the scores of “20,” “40,” “60,” “80,” and “100.” Higher scores indicate greater risk, as shown in Table 2.

### 3.3. Establishment of Risk Indicator Weights

#### 3.3.1. Establishing the Judgment Matrix

Use an appropriate scale to construct a judgment matrix by comparison [26] and establish a comparative judgment matrix A for the risk indicators after statistical analysis:

(1) $$\begin{array}{c} A=\left(aji\right)n\times n=\left(\begin{array}{cccc} a11 & a12 & \cdots & a1n\\ a21 & a22 & \cdots & a2n\\ \vdots & \vdots & \; & \vdots \\ am1 & am2 & \cdots & amn \end{array}\right). \end{array}$$

#### 3.3.2. Calculation of Criterion Layer Weights

The calculation of the weight of the criterion layer can be divided into three steps: one is to normalize the risk judgment matrix A of the criterion layer of the company to obtain a new matrix [27]. The weights are obtained by normalization [28]. The third is the matrix consistency test [29].

(1) Normalize each column of the A matrix to obtain a new matrix *Z*:
  (2) $$\begin{array}{c} Zij=\frac{Aij}{\sum Aij}. \end{array}$$
(2) The eigenvectors are obtained by summing each row of the matrix, and then the weights are obtained by normalizing the eigenvectors:
  (3) $$\begin{array}{c} Wi=\frac{Zi}{\sum Aij}. \end{array}$$
WA = (WA 1, WA 2, WA 3, WA 4, WA 5).
From this, it can be concluded that WA1 to WA5 are the weight ratios of each risk factor index in each criterion layer, and the next work is to take a consistency check on the weight of each index obtained.
(3) Matrix consistency test

We calculate the largest eigenroot as follows:

(4) $$\begin{array}{c} \lambda \max=\frac{\sum \left(AW\right)i}{nWi}. \end{array}$$

where *λ*max represents the largest eigenvalue, *A* represents the corresponding matrix, *W* represents the eigenvector, and *i* represents the corresponding element in the matrix. The CI scale is determined based on the characteristic root. The formula is as follows:

We calculate the consistency index of the judgment matrix as follows:

(5) $$\begin{array}{c} \text{CI}=\frac{\lambda \max-n}{n-1}. \end{array}$$

Factor CR agreement was calculated according to the RI corresponding to the CI. In fact, RI is a constant, which represents the average random consistency index. According to the order of the matrix, the ratio of the matrix consistency index CI and the average random consistency index RI of the same order can be queried in the table, which is called the random consistency ratio. If the condition of CR < 0.10 is satisfied, it can indicate that the judgment matrix has passed the consistency check, and if it is not satisfied, it means that the consistency check has not passed [30].

We calculate the random consistency ratio as follows:

(6) $$\begin{array}{c} \text{CR}=\frac{\text{CI}}{\text{RI}}. \end{array}$$

#### 3.3.3. Calculation of Index Layer Weights and Comprehensive Weights

When determining other weights, you can also collect and analyze data and use the same method as above to calculate the standard layer judgment matrix weight.

According to the formula: the comprehensive weight of the indicator layer = the weight of the indicator layer × the weight of the criterion layer, the comprehensive weight of each indicator of the company's indicator layer can be obtained by calculation.

### 3.4. Application of the Fuzzy Comprehensive Evaluation Method

After the weight of each risk factor index is obtained, the membership degree of the fuzzy comprehensive evaluation set should be calculated next, and the fuzzy comprehensive evaluation should be implemented by combining the weight and the membership degree [31]. The determination of membership degree is highly subjective, requiring each evaluation expert to be careful [32]. The membership matrix function usually refers to a new matrix that is synthesized after the evaluation indicators of all matrices are rated by membership [33], as shown in the following formula:

(7) $$\begin{array}{c} R=\left(\begin{array}{ccc} r11 & \cdots & r1n\\ \vdots & \ddots & \vdots \\ rm1 & \cdots & amn \end{array}\right). \end{array}$$

*R* can be regarded as a mapping of the matrix membership evaluation set, and the membership degree is treated as a condition of fuzzy operation, and the fuzzy evaluation result can be obtained by multiplying it by the weight. The specific calculation formula is shown in the following formula:

(8) $$\begin{array}{c} B=W\cdot R=\left(W1,W2,W3,\ldots ,Wn\right)\cdot \left(\begin{array}{ccc} r11 & \cdots & r\;\ln\\ \vdots & \ddots & \vdots \\ rm1 & \cdots & rmn \end{array}\right). \end{array}$$

Formula (8) can be used to calculate the fuzzy comprehensive evaluation score of the five matrices of the criterion layer “A1” to “A5.” From the above calculation ideas, usually use “very important, relatively important, generally important, less important, very unimportant,” the 5-level satisfaction evaluation level that makes a reasonable evaluation of all evaluation indicators, so as to obtain the membership degree. Twenty experts selected Appendix B and obtained the evaluation frequency table after statistics. The corresponding membership degree matrix can be obtained by obtaining the membership degree of each index.

## 4. Case Validation

### 4.1. Case Situation

HIG bookkeeping company was established in 2013. It is a typical small- and medium-sized bookkeeping company in China. The company has a registered capital of 1 million yuan. Its business scope includes accounting business consulting services, accounting consultants, agency bookkeeping services [34], agency financial and tax reporting services, agent for industrial and commercial registration, enterprise annual report service, agent for various licenses, and agent for trademark registration and patent application [35].

After the discussion of 20 experts, the final conclusion is drawn to the HIG company's agency bookkeeping risk formation table, as shown in Table 3.

### 4.2. Establishment of Risk Factor Indicator Weights

#### 4.2.1. Constructing the Judgment Matrix

A total of 20 experts were invited for this case, including 3 managers and deputy managers of the company; one person in charge of each department of Administration Department, Operation Department, Business Department, and Finance Department; and 13 external financial experts. After statistical analysis, a comparison (judgment) matrix A is established for the risk indicators:

(9) $$\begin{array}{c} A=\left(aji\right)n\times n=\left(\begin{array}{cccc} a11 & a12 & \cdots & a1n\\ a21 & a22 & \cdots & a2n\\ \vdots & \vdots & \; & \vdots \\ am1 & am2 & \cdots & amn \end{array}\right),\\ A=\left(\begin{array}{ccccc} 1 & 4 & \frac{1}{2} & 3 & \frac{1}{3}\\ \frac{1}{4} & 1 & \frac{1}{4} & \frac{1}{3} & \frac{1}{4}\\ 2 & 4 & 1 & 3 & \frac{1}{2}\\ \frac{1}{3} & 3 & \frac{1}{3} & 1 & \frac{1}{5}\\ 3 & 4 & 2 & 5 & 1 \end{array}\right). \end{array}$$

#### 4.2.2. Calculation of Criterion Layer Weights

(1) Normalize each column of the *A* matrix to obtain a new matrix *Z* as follows:
  (10) $$\begin{array}{c} Zij=\frac{Aij}{\sum Aij},\\ Z=\left(\begin{array}{ccccc} 0.15 & 0.25 & 0.12 & 0.24 & 0.15\\ 0.04 & 0.06 & 0.06 & 0.03 & 0.11\\ 0.30 & 0.25 & 0.24 & 0.24 & 0.22\\ 0.05 & 0.19 & 0.08 & 0.08 & 0.09\\ 0.46 & 0.25 & 0.49 & 0.41 & 0.44 \end{array}\right). \end{array}$$
(2) The eigenvectors are obtained by summing each row of the matrix, and then the weights are obtained by normalizing the eigenvectors [36]:
  (11) $$\begin{array}{c} Wi=\frac{Zi}{\sum Aij}. \end{array}$$
WA = (WA 1, WA 2, WA 3, WA 4, WA 5) = (0.1827, 0.0596, 0.2522, 0.0977, 0.4078).
(3) Matrix consistency test

We calculate the largest eigenroot as follows:

(12) $$\begin{array}{c} \lambda \max=\frac{\sum \left(AW\right)i}{nWi}. \end{array}$$

Here, *λ*max = 5.2541.

We calculate the consistency index of the judgment matrix as follows:

(13) $$\begin{array}{c} CI=\frac{\lambda \max-n}{n-1}. \end{array}$$

Here, *CI* = 0.0635.

The average random consistency index is shown in Table 4.

We calculate the random consistency ratio as follows:

(14) $$\begin{array}{c} \text{CR}=\frac{\text{CI}}{\text{RI}}. \end{array}$$

H CR = 0.0567 < 0.10.

Therefore, it can be determined that WA = (0.1827, 0.0596, 0.2522, 0.0977, 0.4078) is the criterion layer weight that satisfies the consistency test conditions.

#### 4.2.3. Calculation of Indicator Layer Weights

Using the same method as above, the standard layer judgment matrix weights are calculated as shown in Tables 5–9, respectively.

*λ*max = 3.0735 and CR = 0.0707 < 0.10.

Indicator layer weights for policy legal risks: WA1 = (0.1717, 0.4414, 0.3869).

*λ*max = 3.0037 and CR = 0.0036 < 0.10.

The indicator layer weight of industry competition risk: WA2 = (0.0994, 0.3736, 0.5270).

*λ*max = 3.0015 and CR = 0.0014 < 0.10.

Indicator layer weights for information technology risk: WA3 = (0.6300, 0.1515, 0.2185).

*λ*max = 4.1315 and CR = 0.0493 < 0.10.

Indicator layer weights for undertaking business risks: WA4 = (0.2664, 0.0840, 0.5083, 0.1413).

*λ*max = 4.1471 and CR = 0.0551 < 0.10.

The weight of the practitioner risk indicator layer: WA5 = (0.5325, 0.2542, 0.0911, 0.1222).

#### 4.2.4. Calculation of Comprehensive Weight of Index Layer

According to the formula: the comprehensive weight of the indicator layer = the weight of the indicator layer × the weight of the criterion layer, the comprehensive weight of each indicator in the indicator layer of HIG can be obtained by calculation, as shown in Table 10.

It can be found from Table 10 that the top three comprehensive weights of the indicator layer are professional skills risk, financial software technology risk, and professional ethics risk.

### 4.3. Application of the Fuzzy Comprehensive Evaluation Method

#### 4.3.1. Establishment of the Membership Matrix

Twenty experts selected Appendix B and obtained the evaluation frequency table after statistics, as shown in Table 11.

Taking the membership evaluation of a11 as an example, it is very important for 2 experts to choose a11; the choice of 8 experts is more important; the choice of 8 experts is generally important; the choice of 2 experts is not very important; and the choice of no experts is very unimportant. Then the membership degree of a11 is as follows: r11 = (0.1, 0.4, 0.4, 0.1, 0), and so on, the corresponding membership degree matrix can be obtained by obtaining the membership degree of each index.

(15) $$\begin{array}{c} R1=\left(\begin{array}{ccccc} 0.1 & 0.4 & 0.4 & 0.1 & 0\\ 0.2 & 0.4 & 0.3 & 0.1 & 0\\ 0.1 & 0.3 & 0.4 & 0.2 & 0 \end{array}\right),\\ R2=\left(\begin{array}{ccccc} 0.1 & 0.2 & 0.5 & 0.1 & 0.1\\ 0 & 0.3 & 0.5 & 0.1 & 0.1\\ 0.1 & 0.1 & 0.5 & 0.2 & 0.1 \end{array}\right),\\ R3=\left(\begin{array}{ccccc} 0 & 0.3 & 0.2 & 0.1 & 0.1\\ 0.1 & 0.4 & 0.3 & 0.2 & 0\\ 0.1 & 0.3 & 0.4 & 0.2 & 0 \end{array}\right),\\ R4=\left(\begin{array}{ccccc} 0 & 0.3 & 0.4 & 0.2 & 0.1\\ 0.1 & 0.3 & 0.4 & 0.1 & 0.1\\ 0.1 & 0.4 & 0.4 & 0.2 & 0\\ 0 & 0.3 & 0.4 & 0.2 & 0.1 \end{array}\right),\\ R5=\left(\begin{array}{ccccc} 0.1 & 0.4 & 0.4 & 0.1 & 0\\ 0.1 & 0.3 & 0.4 & 0.2 & 0\\ 0 & 0.3 & 0.5 & 0.2 & 0\\ 0.1 & 0.2 & 0.5 & 0.1 & 0.1 \end{array}\right),\\ R=\left(\begin{array}{ccccc} 0.2 & 0.3 & 0.4 & 0.1 & 0\\ 0.1 & 0.3 & 0.4 & 0.2 & 0\\ 0.2 & 0.3 & 0.4 & 0.1 & 0\\ 0.2 & 0.2 & 0.4 & 0.2 & 0\\ 0.1 & 0.3 & 0.5 & 0.1 & 0 \end{array}\right). \end{array}$$

#### 4.3.2. Fuzzy Operations

Taking the criterion-level indicator of policy and legal risk as an example, according to formula (8), its membership algorithm is

(16) $$\begin{array}{c} B=W1\cdot R1=\left(0.1717,0.4414,0.3569\right)\cdot \left(\begin{array}{ccccc} 0.1 & 0.4 & 0.4 & 0.1 & 0\\ 0.2 & 0.4 & 0.3 & 0.1 & 0\\ 0.1 & 0.3 & 0.4 & 0.2 & 0 \end{array}\right). \end{array}$$

 
*B*1 = (0.1411, 0.3523, 0.3439, 0.1327, 0)
  The same can be obtained:
 
*B*2 = (0.0626, 0.1847, 0.5, 0.1527, 0.1)
 
*B*3 = (0.226, 0.3151, 0.2589, 0.137, 0.063)
 
*B*4 = (0.0592, 0.3508, 0.4, 0.1916, 0.0492)
 
*B*5 = (0.0909, 0.341, 0.4213, 0.1345, 0.0122)
  Normalized to get:
 
*B*1 = (0.1455, 0.3632, 0.3545, 0.1368, 0)
 
*B*2 = (0.0626, 0.1847, 0.5, 0.1527, 0.1)
 
*B*3 = (0.226, 0.3151, 0.2589, 0.137, 0.063)
 
*B*4 = (0.0563, 0.3338, 0.3807, 0.1823, 0.0468)
 
*B*5 = (0.0909, 0.341, 0.4213, 0.1345, 0.0122)
  Target layer fuzzy evaluation results:
 
*B* = W·R = (0.1533, 0.2902, 0.4408, 0.1157, 0)

Using the corresponding scores of the previous evaluation set, the risk scores of each factor can be obtained by operation:

 
*B*1 = 0.1455 × 20 + 0.3632 × 40 + 0.3545 × 60 + 0.1368 ×  80 = 49.65
 
*B*2 = 0.0626 × 20 + 0.1847 × 40 + 0.5 × 60 + 0.1527 ×  80 + 0.1 × 100 = 60.86
 
*B*3 = 0.226 × 20 + 0.3151 × 40 + 0.2589 × 60 + 0.137 ×  80 + 0.063 × 100 = 49.92
 
*B*4 = 0.0563 × 20 + 0.3338 × 40 + 0.3807 × 60 +  0.1823 × 80 + 0.0468 × 100 = 56.58
 
*B*5 = 0.0909 × 20 + 0.341 × 40 + 0.4213 × 60 + 0.1345 ×  80 + 0.0122 × 100 = 52.72
 
*B* = 0.1533 × 20 + 0.2902 × 40 + 0.4408 × 60 + 0.1157 ×  80 = 50.38

### 4.4. Analysis of Risk Assessment Results

From the results of the fuzzy comprehensive evaluation, the influence of each risk factor in the criterion layer can be comprehensively analyzed; the degree of attention to the risk factors can be determined; and corresponding countermeasures can be formulated. Finally, analyze the main risk factors, focus on the top three risk factors ranked by the comprehensive weight of the indicator layer, and focus on the response.

## 5. Discussion

The main research methods of this study are the analytic hierarchy process and the fuzzy comprehensive evaluation method. Analytic hierarchy process is a decision analysis method that combines qualitative and quantitative analysis to solve complex multiobjective problems; the relative importance of each decision-making scheme is given; the weight of each standard of each decision-making scheme is reasonably given; and the weights are used to obtain the superior and inferior order of each scheme, which can be effectively applied to those problems that are difficult to solve by quantitative methods. The fuzzy comprehensive evaluation method is a comprehensive evaluation method that transforms qualitative evaluation into quantitative evaluation through the membership degree theory of fuzzy mathematics. The above two methods are greatly influenced by personal subjectivity, have certain limitations, and need to be improved.

## 6. Conclusions

There are now few small- and medium-sized bookkeeping firms, and the industry's future prospects are unclear. Future social and economic development are inextricably linked to long-term sustainable development. As a result, there are fewer studies on these organisations that are relevant, and risk management studies are more beneficial. This study uses an analytic hierarchy process and a fuzzy comprehensive assessment approach to successfully combine quantitative and qualitative analysis and create a multilevel analysis structure model of the risk management evaluation index system of small- and medium-sized agency accounting firms. The specific risk score of each factor is calculated through the scores of 20 experts, and the importance of risk is judged according to the size of the score, which helps the company formulate corresponding risk measures. This research provides a reference for the risk management of enterprises in this industry and has certain research value.

## Figures and Tables

**Figure 1:** Comprehensive risk management framework.

**Figure 2:** Five steps to comprehensive risk management.

**Figure 3:** Formation diagram of agency bookkeeping risk.

**Figure 4:** The specific step of the analytic hierarchy process.

**Figure 5:** The specific step of the fuzzy comprehensive evaluation method.

**Table 1:** Risk evaluation index system.

Target layer	Criterion layer	Indicator layer
Risk assessment influencing factors A of small- and medium-sized bookkeeping companies	Policy and legal risk A1	Industry policy risk a11
		Legal and regulatory risks a12
		Industry regulatory risk a13
	Industry competition risk A2	Risk a21 of low-price competition among peers
		Infiltrator substitution risk a22
		Service homogenization risk a23
	Information technology risk A3	Financial software technology risk a31
		Financial data access risk a32
		Internal information process risk a33
	Undertaking business risk A4	Delegator moral hazard a41
		Risk a42 of loss of customer data
		Accounting information distortion risk a43
		Service charge recovery risk a44
	Practitioner risk A5	Professional skills risk a51
		Professional ethics hazard a52
		Employee training risk a53
		Liquidity risk a54

**Table 2:** Risk assessment level.

Risk level	Evaluation results	Evaluation scores
1	No risk	20
2	Small risk	40
3	Average risk	60
4	High risk	80
5	Huge risk	100

**Table 3:** Risk formation table of HIG's agency bookkeeping.

Risk factor	Possible risk events	Risk taker	Risk loss
Policy and legal risks	Inadequate state support for the industry	HIG company	Loss of business development
	Contractual dispute	HIG company	Loss of business management
	Irregularities in the industry	HIG company	Loss of business development
Industry competition risk	Industry price disorder	HIG company	Loss of business development
	Market share is seized by newcomers	HIG company	Loss of business development
	No competitive advantage	HIG company	Loss of business development
Information technology risk	Intelligent financial software	HIG company	Loss of business development
	Loss of financial data	HIG company	Loss of service quality
	Poor communication of internal information	HIG company	Loss of business management
Undertaking business risk	Principal's tax evasion	HIG company	Loss of business management
	Loss of customer data	HIG company, Entrusting company	Loss of service quality
	Distortion of accounting information	HIG company, Entrusting company	Loss of service quality
	Not received service fee	HIG company	Loss of business management
Practitioner risk	Unprofessional staff	HIG company	Loss of service quality
	The moral quality of the employees is not high, and they make false accounts	HIG company	Loss of service quality
	Employee training is not appropriate, or if they learn skills, they will leave	HIG company	Loss of labor costs
	Resign after being familiar with the operation process, revealing business opportunities	HIG company	Loss of business talent

**Table 4:** Mean random consistency indicator.

Order, *n*	1	2	3	4	5	6	7	8	9
RI	0	0	0.52	0.89	1.12	1.26	1.36	1.41	1.46

**Table 5:** The scoring results of the policy and legal risk indicator layer.

Policy and legal risk A1	Industry policy risk a11	Legal and regulatory risks a12	Industry regulatory risk a13	Wi
Industry policy risk a11	1	1/2	1/3	0.1717
Legal and regulatory risks a12	2	1	3/2	0.4414
Industry regulatory risk a13	3	2/3	1	0.3869

**Table 6:** The scoring results of the industry competition risk index layer.

Industry competition risk A2	Risk a21 of low-price competition among peers	Infiltrator substitution risk a22	Service homogenization risk a23	Wi
Risk a21 of low-price competition among peers	1	1/4	1/5	0.0994
Infiltrator substitution risk a22	4	1	2/3	0.3736
Service homogenization risk a23	5	3/2	1	0.5270

**Table 7:** The scoring results of the information technology risk index layer.

Information technology risk A3	Financial software technology risk a31	Financial data access risk a32	Internal information process risk a33	Wi
Financial software technology risk a31	1	4	3	0.6300
Financial data access risk a32	1/4	1	2/3	0.1515
Internal information process risk a33	1/3	3/2	1	0.2185

**Table 8:** The scoring results of the indicator layer for undertaking business risks.

Undertaking business risk A4	Delegator moral hazard a41	Risk a42 of loss of customer data	Accounting information distortion risk a43	Service charge recovery risk a44	Wi
Delegator moral hazard a41	1	3	1/3	3	0.2664
Risk a42 of loss of customer data	1/3	1	1/5	1/2	0.0840
Accounting information distortion risk a43	3	5	1	3	0.5083
Service charge recovery risk a44	1/3	2	1/3	1	0.1413

**Table 9:** Scoring results at the practitioner risk indicator layer.

Practitioner risk A5	Professional skills risk a51	Professional ethics hazard a52	Employee training risk a53	Liquidity risk a54	Wi
Professional skills risk a51	1	3	4	5	0.5325
Professional ethics hazard a52	1/3	1	3	3	0.2542
Employee training risk a53	1/4	1/3	1	1/2	0.0911
Liquidity risk a54	1/5	1/3	2	1	0.1222

**Table 10:** The comprehensive weight of the indicators of the HIG company's indicator layer.

Index	Policy and legal risk A1	Industry competition risk A2	Information technology risk A3	Undertaking business risk A4	Practitioner risk A5	The comprehensive weight of the indicator layer	Rank the top three
	0.1827	0.0596	0.2522	0.0977	0.4078		
Industry policy risk a11	0.1717					0.0314	
Legal and regulatory risks a12	0.4414					0.0806	
Industry regulatory risk a13	0.3869					0.0707	
Risk a21 of low-price competition among peers		0.0994				0.0059	
Infiltrator substitution risk a22		0.3736				0.0223	
Service homogenization risk a23		0.5270				0.0314	
Financial software technology risk a31			0.6300			0.1589	2
Financial data access risk a32			0.1515			0.0382	
Internal information process risk a33			0.2185			0.0551	
Delegator moral hazard a41				0.2664		0.0260	
Risk a42 of loss of customer data				0.0840		0.0082	
Accounting information distortion risk a43				0.5083		0.0497	
Service charge recovery risk a44				0.1413		0.0138	
Professional skills risk a51					0.5325	0.2171	1
Professional ethics hazard a52					0.2542	0.1037	3
Employee training risk a53					0.0911	0.0371	
Liquidity risk a54					0.1222	0.0498	

**Table 11:** Statistical table of frequency of satisfaction evaluation of five levels of risk factors.

Risk factor	Very important	Relatively important	Generally important	Less important	Very unimportant
	Frequency	Frequency	Frequency	Frequency	Frequency
Policy and legal risk A1	4	6	8	2	0
Industry policy risk a11	2	8	8	2	0
Legal and regulatory risks a12	4	8	6	2	0
Industry regulatory risk a13	2	6	8	4	0
Industry competition risk A2	2	6	8	4	0
Risk a21 of low-price competition among peers	2	4	10	2	2
Infiltrator substitution risk a22	0	6	10	2	2
Service homogenization risk a23	2	2	10	4	2
Information technology risk A3	4	6	8	2	0
Financial software technology risk a31	6	6	4	2	2
Financial data access risk a32	2	8	6	4	0
Internal information process risk a33	2	6	8	4	0
Undertaking business risk A4	4	4	8	4	0
Delegator moral hazard a41	0	6	8	4	2
Risk a42 of loss of customer data	2	6	8	2	2
Accounting information distortion risk a43	2	8	8	4	0
Service charge recovery risk a44	0	6	8	4	2
Practitioner risk A5	2	6	10	2	0
Professional skills risk a51	2	8	8	2	0
Professional ethics hazard a52	2	6	8	4	0
Employee training risk a53	0	6	10	4	0
Liquidity risk a54	2	4	10	2	2

**Table 12:** Criterion level scoring form.

Scale	Definition	Instruction
1	Equally important	The *M* metric is as important as the *N* metric
2		Importance is between 1 and 3
3	Slightly important	The *M* index is slightly more important than the *N* index
4		The importance is between 3 and 5
5	Obviously important	The *M* index is significantly more important than the *N* index
6		The importance is between 5 and 7
7	Much more important	*M* index is much more important than the *N* index
8		The importance level is between 7 and 9
9	Extremely important	*M* index is extremely important than *N* index

Note: if the ratio of the *M* index to the *N* index is *a*, then the ratio of the *N* index to the *M* index is 1/*a*.

**Table 13:** Scoring table of policy and legal risk indicator layer.

Policy and legal risk A1	Industry policy risk a11	Legal and regulatory risks a12	Industry regulatory risk a13
Industry policy risk a11	1		
Legal and regulatory risks a12		1	
Industry regulatory risk a13			1

**Table 14:** Scoring table of industry competition risk indicator layer.

Risk assessment A	Policy and legal risk A1	Industry competition risk A2	Information technology risk A3	Undertaking business risk A4	Practitioner risk A5
Policy and legal risk A1	1				
Industry competition risk A2		1			
Information technology risk A3			1		
Undertaking business risk A4				1	
Practitioner risk A5					1

Industry competition risk A2	Risk a21 of low-price competition among peers	Infiltrator substitution risk a22	Service homogenization risk a23		
Risk a21 of low-price competition among peers	1				
Infiltrator substitution risk a22		1			
Service homogenization risk a23			1		

**Table 15:** Scoring table for the information technology risk indicator layer.

Information technology risk A3	Financial software technology risk a31	Financial data access risk a32	Internal information process risk a33
Financial software technology risk a31	1		
Financial data access risk a32		1	
Internal information process risk a33			1

**Table 16:** Scoring table for the risk indicator layer of undertaking business.

Undertaking business risk A4	Delegator moral hazard a41	Risk a42 of loss of customer data	Accounting information distortion risk a43	Service charge recovery risk a44
Delegator moral hazard a41	1			
Risk a42 of loss of customer data		1		
Accounting information distortion risk a43			1	
Service charge recovery risk a44				1

**Table 17:** Scoring table for practitioner risk indicator tiers.

Practitioner risk A5	Professional skills risk a51	Professional ethics hazard a52	Employee training risk a53	Liquidity risk a54
Professional skills risk a51	1			
Professional ethics hazard a52		1		
Employee training risk a53			1	
Liquidity risk a54				1

**Table 18:** Risk factor membership questionnaire.

Risk factor	Very important	Relatively important	Generally important	Less important	Very unimportant
Policy and legal risk A1					
Industry policy risk a11					
Legal and regulatory risks a12					
Industry regulatory risk a13					
Industry competition risk A2					
Risk a21 of low-price competition among peers					
Infiltrator substitution risk a22					
Service homogenization risk a23					
Information technology risk A3					
Financial software technology risk a31					
Financial data access risk a32					
Internal information process risk a33					
Undertaking business risk A4					
Delegator moral hazard a41					
Risk a42 of loss of customer data					
Accounting information distortion risk a43					
Service charge recovery risk a44					
Practitioner risk A5					
Professional skills risk a51					
Professional ethics hazard a52					
Employee training risk a53					
Liquidity risk a54					

## Data Availability

The data set can be accessed upon request.

## Appendix

### A. Questionnaire for Risk Assessment Indicators

Using the following Saaty's 1–9 scale values, please rate each risk factor in the risk evaluation index system from Tables 12–17.

### B. Risk Factor Membership Questionnaire

Please use the “✔” symbol to select the importance level of different risk factors (Table 18).
